# Tianxia120: A Multimodal Medical Data Collection Bioinformatic System for Proactive Health Management in Internet of Medical Things

**DOI:** 10.1155/2020/8828738

**Published:** 2020-09-26

**Authors:** Zihan Jiao, Yindong Xiao, Yanmei Jin, Xinyu Chen

**Affiliations:** ^1^School of Automation Engineering, University of Electronic Science and Technology of China, Chengdu 611731, China; ^2^School of Information and Communication Engineering, University of Electronic Science and Technology of China, Chengdu 611731, China

## Abstract

A digital medical health system named Tianxia120 that can provide patients and hospitals with “one-step service” is proposed in this paper. Evolving from the techniques of Internet of Medical Things (IoMT), medical dig data, and medical Artificial Intelligence, the system can systematically promote the change of service status between doctors and patients from “passive mode” to “proactive mode” and realize online service that is similar to offline medical treatment scenarios. The system consists of a patient terminal and a doctor terminal. They can perform online inquiry (through graphic, voice, telephone, video, etc.), electronic prescription, multiparameter self-diagnosis, cold chain logistics, medicine distribution, etc. The system can provide rich medical health information, medical tools browsing, and health care big data aggregation processing functions. Compared with the traditional medical system, this system has the characteristics of full function, rich data, and high security. It is expected to be applied to hospital applications and medical research to promote the construction and innovation of clinical medical disciplines.

## 1. Introduction

The world's population is rapidly aging together with people's increasing concern for healthcare [1]. It is estimated that, by 2050, people aged 60 years and older will reach 2 billion, and 80% of them will live in low- and middle-income countries [2]. In China, for example, the number of elderly people over 60 years old has exceeded 200 million and a large number of people get chronic diseases [3]. And over 90 percent of health care work needs to be carried out by primary health care institutions. However, the level of medical staff in primary health care institutions is uneven. Most patients still prefer top-level hospitals, and this phenomenon has already brought China into an imperative stage to effectively improve national health to a new level [4]. Therefore, the central government of China promulgated the “Healthy China 2030” Planning Outline [5], which is based on the whole population and the whole life cycle to promote the provision of fair and accessible, systematic and continuous health services to achieve a higher level of national health. This situation brings significant opportunities and challenges to the health platform today.

The health platform has been in development for a long time: the Clinical Documentation Architecture (CDA R1) was defined in May 2005 and became the American National Standards Institute (ANSI) approved HL7 standard, which became the specification for the Health Level 7 (HL7) Reference Information Model (RIM) [6]. Although it has been spread around the world, the application is still not extensive enough [7]. The Continuity of Care Document (CCD) is an HL7 CDA implementation of the Continuity of Care Record (CCR). And the CCR data set contains a summary of the patient's health status including problems, medications, allergies, and basic information about health insurance, care documentation, and the patient's care plan [8]. Ekonomou et al. presented a cloud-based healthcare system that provides high levels of security and privacy within a cloud environment, enabling sharing of both health records and the access rights, along the patient pathway in 2011 [9]. RF-MediSys presented an innovative electronic medical record (EMR) system, which can perform medical information sharing and retrieval effectively, and it is accessible via a “smart” medical card [10]. But Deng et al. raised concern about cloud security and privacy in home health systems [11]. Tsai et al. implemented the data leakage prevention scheme to avoid illegal duplication [12]. Pan et al. designed a novel electronic medical record system for regional clinics and health centers in China [13]. Despite all these systems, e-health platforms are still not widely used. The development of the health system platform still faces serious challenges, especially in developing countries [14].

With the development of electronic medical equipment, the formation of online medical systems has become possible [15]. Telemedicine is gradually acceptable to patients [16]. The concept of mobile health has emerged as a key beneficiary of the dual emphasis on technology and an increasing interest in health behavior and data monitoring [17]. Based on the integration of “traditional medicine +” Internet of medical things, big data, artificial intelligence, and other intelligent digital technologies, the world is experiencing a stage transition from the medical health prevention based on traditional evidence-based medicine theory and practice to precise and proactive health management mode. Considering this, a digital medical system named Tianxia120 for proactive health management is proposed in this paper as shown in Figure 1. The Tianxia120 digital medical system includes an intelligent digital hospital platform and a proactive healthcare platform.

The two platform systems interact with each other to conduct doctor-patient interaction around the one-stop service of “medical-drug-test-risk.” For patients, not only can it provide online or offline integration for their individual or family members, which is similar to the online medical treatment scene for visiting the hospital for medical advice, but also it can provide a comprehensive system of disease prevention and health management for the whole family. For hospitals, it is also possible to help the medical departments and staff carry out research and applications of production, education, and research based on the “digital technology+” production and research solutions supported by the system. Taking the application of Tianxia120 as an example, this paper will share the experience of proactive health management application based on the digital technology in four main aspects, “architecture design, platform function, innovation mode, and representative application case,” and explore the precision health care solutions, which can be widespread.

## 2. Digital Medical System Architecture

### 2.1. System Technology Architecture

The Tianxia120 digital medical platform system provides professional, proactive, and continuous health care services, which take patients as the center, and advocates the concept transition from “disease-centered” to “health-centered.” Hospital specialist doctors can provide online consultation and communication services for patients so that the patients can consult doctors without leaving home.

As shown in Figure 2, the Tianxia120 digital medical platform system includes a client terminal for patients and a hospital terminal for doctors. In addition to the service of doctor-patient communication (graphic, voice, telephone, and video), electronic prescription, medical logistics delivery, and the remote intelligent multiparameter self-test functions based on IoMT technology, the client terminal also provides a wealth of medical health information, medical tools browsing, and health care big data aggregation processing function. It can provide solutions for the medical staff to study and research and realize the service of doctors and patients. The doctor terminal has the following functions: Expert studio, electronic prescription, medicine prescription, self-defining scale, single consultation, bed entry, and so on.

### 2.2. System Service Architecture

Figure 3 describes the system architecture that includes the following.

#### 2.2.1. Patients as the Service Enjoying Center

In order to effectively solve the problem of out-of-hospital health care for patients, the Tianxia120 digital medical platform system is a patient-centered service that allows patients to enjoy one-step out-of-hospital follow-up service via smart phone when they are not in the hospital. For example, patients can consult doctors conveniently and quickly with graphic voice/telephone/video, and doctors can issue electronic consultations according to their needs. After the pharmacy pharmacist's trial, the drug is delivered by the medicine cold chain logistics, and the family health file is managed online.

#### 2.2.2. Multiple Disciplinary Teams (MDT) as the Service Providing Center

By the guide of serving patients through MDT, and the principle of serving patients by nurse/home doctor assistant, (hospital or attending) physician and expert, it forms the “Tianxia120 MDT service model” for patients.

#### 2.2.3. Digital Technology as the Service Guaranty Center

With the unique multiparameter monitoring technology of IoMT and the “digital medical technology +” solutions formed by other multitechnology aggregations, the Tianxia120 digital medical platform system can guarantee the complete, continuous, and professional follow-up services for patients outside the hospital.

#### 2.2.4. Expert Studio as the Service Implementation Center

An expert studio consisting of “Nurse/Family Doctor–(Hospital or Indication) Physician–Expert” created on the Tianxia120 digital medical platform system by the experts from top-level hospital constitutes a specific service implementation unit that can provide a digital out-of-hospital follow-up service package to patients for a variety of disease prevention.

### 2.3. Proactive Health Continuous Management Architecture

As shown in Figure 4, proactive health continuous management architecture includes the following:

(1) Three active behaviors of patients
  ① Upload personal medical information actively
  ② Upload medical/physical examination data of immediate family members actively
  ③ Contact a nurse, doctor, or specialist for medical advice actively
(2) Three active behaviors of MDT
  ① Contact patients and provide counseling actively
  ② Remind patients to upload medical/physical data of individuals and immediate family members actively
  ③ Make an appointment with a physician or an expert for the patient actively
(3) Three active behaviors of the Tianxia120 platform
  ① Responds to the feedback promptly and actively
  ② Reminds both patients and expert teams actively after the patient purchases the service package automatically
  ③ Provides technical and operational support actively

From the feedback of actual operation, the proactive health continuous management service of the three-way linkage combination of Tianxia120 can not only provide patients with better medical experience and human emotional concern, but also help medical personnel control and manage their own fragmentation time and provide services for patients in an orderly manner.

### 2.4. System Operation and Information Security Assurance System

System operation and maintenance security system includes application access layer, platform service layer, business logic layer, big data support layer, and data layer, and they are combined with each other (Figure 5).

## 3. Digital Medical System Composition

The Tianxia120 digital medical system mainly includes a digital hospital platform and a digital proactive health platform system.

### 3.1. Digital Hospital Platform

At the doctor terminal, the digital hospital platform of Tianxia120APP includes the following main contents (Figure 6):

(1) The Tianxia120 digital medical system allows a limited quantity of medical resources to provide access to out-of-hospital services for more patients.
Digital hospital platform can not only support remote video, telephone, voice, and graphic communication functions, but also provide hospitals and medical staff with remote out-of-hospital follow-up for patients who are inconvenient or do not need to come to medical institutions. Meanwhile, it can also promote “top-level hospital—basic community medical institution—family” medical joint mode through the expert studio, thus truly achieving the sinking of high-quality medical resources, and allow limited quality medical resources to serve more people.
(2) The Tianxia120 digital medical system can provide research and “digital technology+” solutions for hospitals, departments, and medical staff.
The digital hospital platform can also provide assistance to the research of hospitals/departments/medical staff on production, education, and study:
  ① Intelligent custom scientific research data scale collection system (uploading the scientific data scale designed by the hospital/department to the Tianxia120 digital medical system APP system)
  ② Multiparameter detection and monitoring data collection based on IoMT technology
  ③ Comprehensive treatment of health care big data after desensitizing
  ④ Reapplication and promotion of production and research results
(3) Core function composition
  ① MDT expert studio: it is established by an expert of associate professor title or above, and other health care practitioners such as physicians, nurses, pharmacists, and health managers can apply to join. The number of expert studios is not limited. Each expert studio corresponds to a specific disease, and it can generate out-of-hospital follow-up service team consisting of 1 expert, 1 physician, and 1 nurse/home doctor assistant.
  ② Online and offline services: These mainly include online graphic speech, telephone or video consultation; making an e-prescription as needed; sending medicine by chain logistics after the drug is checked by the pharmacy pharmacist; managing the family health files online.
  ③ Intelligent custom research scale: when carrying out scientific research projects, it is indispensable to collect data for scales. In the past, many data collection works relied on manual collection offline, and the efficiency and effect were limited. The intelligent custom scientific research scale function originally created by the Tianxia120 digital medical system greatly changed the status. The scientific research workers submit the scale document to the platform, and the Tianxia120 platform technology center uploads the scale to the platform system after the “document-technical conversion,” which can easily realize the online and offline combined scale data collection. In this way, the data collected is not only large, but also widely distributed, and the acquisition time period is greatly shortened.

### 3.2. Digital Proactive Health Platform

Digital proactive health platform refers to the intelligent digital active health platform system. The main contents of the Tianxia120's patient terminal are as follows (Figures 2, 7, and 8). The proposed system is capable of detecting electroencephalogram (EEG), electrocardiogram (ECG), blood pressure, blood oxygen saturation, venous blood routine, urine routine, body fat, and weight with great sensitivity and stability:

(1) Online consultation: patients who are inconvenient or do not need to come to a medical institution can use the remote video, telephone, voice, graphic, and text of the smart phone to consult medical staff online.
(2) Intelligent health self-test (Figure 9): intelligent multiparameter detection and monitoring equipment based on IoMT technology enables patients to self-measure blood glucose, total cholesterol, uric acid, electrocardiogram, lung function, blood pressure, urine routine, and other human physiological indicators at any time by using IoMT-enabled biosensors, such as electrochemical sensors and immunoassay sensors. These sensors collect samples from patients' fingertips blood or body fluids through a small sample pad to induce chemical reactions and pass the generated electric current or light signals to micro-controller-unit (MCU) for further computing and storage. The measurement data is consequently uploaded to the digital active health platform via Bluetooth connection or Wi-Fi. The platform system provides real-time storage, analysis, and alarms for different values.
Doctors can quickly access the data when online and consulate and interpret the data. Because the biosensors possess great stability and sensitivity, they can completely meet the testing needs of today's medical market.
(3) Remote pharmacy service: depending on the online consultation, the physician can prescribe an electronic prescription for the returning patient, and the practicing pharmacist will review the prescription. Doctors, pharmacists, and nurses can also remind patients to take medication online, receive feedback information from patients, and pay close attention to patient medication dynamics.
(4) Creation of digital health archives: patients can upload basic information, previous medical treatment, and physical examination data and create digital health archives for the whole family through mobile phones.
(5) Online booking and offline service: if necessary, patients can also make an appointment with the medical staff to check and provide consultation services. At the same time, doctors can also check the patient's online consultation and go to the offline hospital for further examination such as blood routine test, X-ray, CT inspection, and nuclear magnetic resonance.
(6) Architectural advantages of the digital proactive health platform:
  ① The intelligent micromedical equipment kit based on the IoMT provides one-stop service to quickly build stable, reliable, safe, and controllable IoMT applications
  ② The platform supports PB-level data volume and millions of Transaction Per Second (TPS) capabilities, providing massive data storage and access capabilities
  ③ The security checking service, which is to use security testing to help enterprises discover security issues in the security certification, distribution network and communication process of intelligent hardware
  ④ Web Application Firewall (WAF) can protect against the attacks of 0 day, interface spamming, and collisions to ensure data is secure enough
  ⑤ Protect server security with Anker to prevent hackers. Situational awareness discovers potential intrusion and attack threats through machine learning and data modeling
  ⑥ The platform shares data of the National Medical Center through the dedicated VPN encryption channel

## 4. Application in Proactive Health Management

### 4.1. Application Model Innovation

The application innovation model of “Industry, University and Research” based on “Digital Technology+” is to apply the innovation of the Internet, medical Internet of things, artificial intelligence, health care big data, 4 G/5 G, biotechnology, and other technical and medical health institutions, phased and selective integration to the online and offline combined services supported by the Tianxia120 system (Figure 10). And it takes the standardized formatting of health care big data gradually formed by the dynamic service process as the core and promotes and verifies the innovation of production, education, and research of medical and health institutions in order to realize the industrial application of more innovative health and medical fields promotion. It collaborates with innovation through online and offline deep integration, develops new technologies and methods, and scientifically realizes clinical transformation to jointly address the global burden of disease and health challenges and benefit global patients.

The core of Tianxia120 “Digital Technology+” production and research application innovation model is health care big data solution, and its main contents are as shown in Figure 11:

#### 4.1.1. Health Care Big Data Collection

It implements data collection through the Tianxia120 smart digital active health medical platform and data exchange collection and sharing management system, including Tianxia120APP patient terminal, doctor terminal, and intelligent custom scientific data acquisition system.

#### 4.1.2. Data Collection and Operation

(1) The past medparagical health file data of patient/family
  ① Users can upload their own/family history medical data through the Tianxia120 client terminal actively or after being reminded by medical staff, including but not limited to CT, nuclear magnetic resonance, X-ray film, ultrasound, and other image examinations and text reports, medical reports, or test samples.
  ② Users can enter the “Health File” to operate easily through the Tianxia120 client terminal.
  ③ Medical staff can also log into the Tianxia120 APP doctor's terminal and enter the “bedside entry” to easily and conveniently collect health medical data from thousands of patients.
(2) Patients/families can monitor data remotely
Through the “Intelligent Self-Test” function of the Tianxia120 client terminal, users can detect and monitor a variety of health care data at home (requires matching intelligent medical equipment). And users manually upload the test data in the hospital including lung function, ECG, blood pressure, blood sugar, urine routine, cholesterol, uric acid, liver function, kidney function, and blood routine. The data is automatically saved after uploading. Every month, the Tianxia120 system automatically forms a health report and sends it to users.
  ① Intelligent self-test process: enter the “Health File” of the Tianxia120 client terminal and add the detection item, and click “Smart Self-Test”; And medical staff can log into the Tianxia120 doctor terminal, enter the “Bedside Entry” to add the detection item, click “Smart Self-test,” and follow the prompts.
  ② Manual uploading process: enter the “Health File” of the Tianxia120 client terminal and add the detection item, and click “Manual Input”; and medical staff can log into the Tianxia120APP doctor terminal, enter the “Bedside Entry” to add the detection item, click “Manual Input,” and follow the prompts.
  ③ Health self-test process: enter the “Health File” of the Tianxia120 client terminal and click “Health Self Test”; medical staff can log into the Tianxia120 doctor terminal to enter the “bedside entry,” click “Health Self Test,” and follow the prompts.
    1. Patients' network consultation data includes data generated by out-of-hospital follow-up service package consultation, data generated by online single consultation, and data generated by free consultation.
    2. The medication data of patients/family members include the prescription record data issued in the hospital uploaded by patients/family members, electronic prescription records of common diseases, and chronic diseases prescribed by the doctor of the Tianxia120 platform within the limits of regulations.

#### 4.1.3. Health and Medical Big Data Cleaning (Figure 12)

According to the needs of scientific research projects, the data should be cleaned based on Tianxia120 big data Extract-Transform-Load (ETL) cleaning and finishing technology. The process is as follows (Figure 13):

1. Unified data standardization processing
2. Unified description and storage management, unified modeling of various data items
3. ETL operations such as cleaning, verification, and desensitization of big data warehouses

#### 4.1.4. Analysis and Visualization Application of Health Medical Big Data

Relying on the big data analysis and visualization technology of Tianxia120 health care, the research data that has been clearly sorted should be mined, analyzed, and visualized application:

1. Data preparation-multipath association multidatabase table
2. Data multidimensional analysis-multidimensional index database search and retrieval analysis of big data according to scientific research projects
3. Data visualization report rendering-Computer-side browser URL view visualization report/export to excel report program report view

### 4.2. Results of Application Cases

1. Multiple biochemical data collected by the Tianxia120 digital medical system can be used by the study of chronic disease management [18–22].
2. The key research project of the Sichuan Provincial Health Planning Commission “Leshan People's Hospital: Research on the Construction Model of Digital Medical Integration and Demonstration Ward” has applied the Tianxia120 digital medical system to provide many patients for “in-hospital and out-hospital” digital medical services in Leshan downtown and surrounding areas.
3. The key research project of Sichuan Province--“Neijiang First People's Hospital: Application Research on Regional Platform Management Mode of Family Doctor Contracting Service Using “Internet +”” is also applying Tianxia120 digital medical system to provide many patients for “in-hospital and out-hospital” digital medical services in Leshan downtown and surrounding areas.
4. The project that won the second prize of Sichuan Science and Technology Progress Award in 2018--<West China second prize of Sichuan University: Aging and aging function promote innovative research and transformation of results> is also based on the Tianxia120 digital medical system, and provides “prehospital, in-hospital, and posthospital” intelligent medical care and new technology for elderly patients.
5. The digital out-of-hospital follow-up service created by Tianxia120 Digital Medical System has been applied in dozens of large-scale hospitals in China, such as West China Hospital of Sichuan University, the First Affiliated Hospital of Nanchang University, the Second Affiliated Hospital of Nanchang University, the People's Hospital of Leshan City, the First People's Hospital of Neijiang City, the Third Affiliated Hospital of Guangzhou Medical University, etc.
6. For patients, the digital outpatient follow-up proactive health service model of “Third-level hospitals-grassroots community medical institutions-families (individuals)” built by Tianxia120 digital medical system can not only provide online and offline integration for its individual or family members, which is similar to the online medical treatment scene for visiting the hospital for medical advice, but also provide a comprehensive system of disease prevention and health management for the whole family. For hospitals, it can also help hospitals/departments manage patients by disease based on system-supported “digital technology+” production and research solutions. By managing patients through mobile phones and collecting scientific research data, it can help hospitals, departments, and medical staff to carry out research data and application of production, education, and research to promote the construction and innovation of clinical medicine disciplines and the empowerment of hospitals.

## Figures and Tables

**Figure 1:** System technology architecture.

**Figure 2:** The Tianxia120 digital medical system.

**Figure 3:** System service architecture.

**Figure 4:** Proactive health continuous management architecture.

**Figure 5:** System operation and information security assurance system.

**Figure 6:** Technical architecture.

**Figure 7:** Business structure.

**Figure 8:** Technical framework.

**Figure 9:** Intelligent multiparameter detection and monitoring device based on Internet of Medical Things (IoMT) technology application.

**Figure 10:** The Architecture of the application innovation model of “Industry-University-Research,” which is based on “Digital Technology+.”

**Figure 11:** Technical framework health medical big data system.

**Figure 12:** Demonstration of medical big data cleaning process.

**Figure 13:** Process of health care big data analysis and visualization.

## Data Availability

All data used during the study are available from the corresponding author upon request.
